The article "Paradigm and Path of Released Prisoners' Rights of Rehabilitation from the Perspective of Social Governance" was retracted in 2023. Reasons: unreliable results or conclusions; concerns about the data; concerns about the peer review; concerns about the citations.

# Paradigm and Path of Released Prisoners' Rights of Rehabilitation from the Perspective of Social Governance

**DOI:** 10.1155/2022/6266082

**Published:** 2022-09-19

**Authors:** Meifeng Ma

**Affiliations:** School of Law, Politics, Economy and Trade, Chongqing University of Science and Technology, Chongqing 401331, China

## Abstract

In order to better solve the problem of the return of released prisoners to society and reduce the second crime rate after rehabilitation, the main factors affecting the rehabilitation of released prisoners and the specific situation of reoffending were studied from the perspective of social governance. There is a big difference between the sentence period of the first crime and the second crime. The proportion of those sentenced to less than 5 years for the first time is 86.1%, and the proportion of those sentenced to less than 3 years for the second time is 31.1%. Compared with the first crime, the proportion of those sentenced to more than 10 years has decreased by 56.7%, and the proportion of those sentenced to more than 10 years has increased by 8.6%. The figure shows that second offenses are more serious than first offenses. Those released from prison are likely to commit crimes again at any time after rehabilitation, and the proportion of reoffending within 5 years is 73.3%. The proportion of reoffenders who committed crimes for more than 5 years was 26.7%, indicating that the 5-year period after rehabilitation should be taken seriously to reduce the second crime rate. On this basis, the countermeasures for the rehabilitation of released prisoners are discussed.

## 1. Introduction

As a special group in the social group, a person released after serving his sentence is punished by the law because he has violated the law. After being pronounced by the court, the criminal law enforcement organ carries out the punishment according to law, and after a certain period of prison reform, he is released according to law [1]. The reason why this group is special is that after having criminal experience and returning to society, most of them have low education levels, no education background, no professional skills, no job, unstable economic sources, no income, and so on. For those released from prison, it is inevitable that there will be some alternative views or prejudice and discrimination in society. In addition, the punishment imposed by the law on those released from prison reflects that most of them have failed to receive education since childhood. In other words, the failure of the initial socialization, after the release from prison, is undoubtedly difficult to return to society, and the difficulty of resocialization will be even greater. The working and living conditions of released persons after their return to society are the basis for promoting the formulation and improvement of relevant public policies.

The article "Paradigm and Path of Released Prisoners' Rights of Rehabilitation from the Perspective of Social Governance" was retracted in 2023. Reasons: unreliable results or conclusions; concerns about the data; concerns about the peer review; concerns about the citations.

After serving their sentences, the released persons must face the problem of how to recover their rights and how to return to society, which is a relatively difficult process. According to a large number of investigations, the living conditions of most released prisoners after their return to society are not very optimistic, so it has gradually become a social problem of universal concern. In the process of promoting the healthy development of social governance, we must build a good mechanism to solve these problems. From an academic point of view, released prisoners are vulnerable groups in terms of social survival, as well as dangerous groups. Therefore, great attention must be paid to social affairs, social adaptation, and social protection of these people after their rights are restored. How to overcome the difficulties in employment, marriage, family, and interpersonal communication after the release of prison term is the focus of this study, so as to turn passivity into the initiative and reduce the probability of committing crimes again [2].

With the concern of this problem, China's resettlement, help, education, and protection work have been carried out rapidly in the whole country and have made some achievements, but there is still a big gap compared with overseas developed countries and regions [3]. Their restoration protection system was established earlier and constantly improved in practice, but China's penalty concept and economic status are still relatively backward; these seriously restrict the development of restoration protection work, and there are still many places to solve this problem.

## 2. Literature Review

From the perspective of social adaptation, Wang et al. believed that the life course of released prisoners experienced at least two adaptation processes: the first adaptation was the adaptation from the social system to the prison system and the second is release from the prison system to the social system. In modern society, any individual's behavior requires advice, help, and guidance of professionals [4]. Romano et al. believe that in such a modern, complex, and complicated society (Figure 1), individuals or groups increasingly believe in professional knowledge. Before doing anything, they always refer to various professional opinions and find the basis for behavior. Without professional knowledge, individuals will be at a loss [5]. The ex-convicts are a group of people who do not have the expertise, and the society that they live in before they are released and the society that they live in after they are released are very different [6].

The article "Paradigm and Path of Released Prisoners' Rights of Rehabilitation from the Perspective of Social Governance" was retracted in 2023. Reasons: unreliable results or conclusions; concerns about the data; concerns about the peer review; concerns about the citations.

Through their research, Mees and Smith found that social integration not only includes the exclusion conflict between different groups and ordinary groups but also includes the gradual dissolution of the exclusion conflict between the two groups and then the process of mutual adaptation, mutual identification, and mutual integration [7]. The research of Borzel et al. found that in the dimension of economic integration, the degree of integration of those with employment intention is higher than that of those without employment intention. The degree of integration of the strong desire to communicate with others is higher than that of the weak desire to communicate with others. The integration degree of people with social insurance is higher than that of people without social insurance. Employers do not take the political audit as the hiring standard to change the degree of group integration is higher [8]. In the dimension of cultural integration, those who are willing to communicate with others have a higher degree of integration than those who are unwilling to communicate with others. Employers do not take the political examination as the recruitment standard; the group integration degree is higher. Huang and Chen found that in the dimension of social relationship integration, the degree of integration of people with higher education is higher than that of people with lower education. The degree of integration of the strong desire to communicate with others is higher than that of the weak desire to communicate with others. In terms of the overall level of social integration, the integration degree of those with higher education levels is higher than that of those with lower education levels. The degree of integration of the strong desire to communicate with others is higher than that of the weak desire to communicate with others. Employers do not take the political examination as the admission standard; the group integration degree is higher [9]. Different from domestic scholars' emphasis on the significance of recidivism and social adaptation of released prisoners to society, foreign scholars emphasize considering their return to society from the micro level of their own psychology, change of situation, daily life, and so on.

Karatal et al. believe that the social adjustment process of released prisoners can be divided into the excitement period, sobriety period, and reorientation period. When released from prison, ex-convicts are excited about being free again; they want to do a lot of things they could not do because of being in prison. They are eager to turn over a new leaf and make up their lost time. It is also a time when families are excited to see ex-prisoners again and encourage them eagerly. This is called the euphoric period [10]. Rodríguez-Fernández et al. have looked at turning points in behavior change over the course of life. By exploring whether work is a turning point in the life course of offenders and whether criminals stop committing crimes if they have a job, it is concluded that age and employment interact to affect self-reported recidivism rates. People aged 27 or older are less likely to commit crimes or be arrested when marginal employment opportunities are offered than when they are not [11].

The article "Paradigm and Path of Released Prisoners' Rights of Rehabilitation from the Perspective of Social Governance" was retracted in 2023. Reasons: unreliable results or conclusions; concerns about the data; concerns about the peer review; concerns about the citations.

## 3. Released Persons Return to the Status Quo of Social Cooperation and Governance

### 3.1. The Basic Situation of the Persons Released after Serving Their Sentence in China

Except for a small number of criminals sentenced to death, the vast majority of criminals will eventually return to society after education and reform [12]. The author has defined the scope of this study as prison-released persons. The statistics made by the Ministry of Justice on prison-released persons in recent years is summarized in Figure 2

As can be seen from the data and growth trend in Figure 2, except in 2012, the number of released prisoners decreased slightly, and then it continued to increase. Although there is no statistics on the number of people released from prison in 2016, the trend is that the number will be higher than that in 2015. The increase in number will inevitably lead to more and more people facing the problem of returning to society. In fact, a considerable number of people released from prison will lead a very difficult life for a certain period of time after their release [13].

### 3.2. The Social Protection of the Released Persons in China

#### 3.2.1. The Integration of Released Persons with Society

In 2015, resettlement, help, and education organizations at all levels connected about 806,800 people released after serving their sentences, of which 363,700 were connected to prisons, accounting for only 69.1 of the total number. In 2014, 736,200 people were transferred to prisons after serving their sentences, of whom 351,900 were released from prisons, accounting for 71.08% of the total number. In 2013, there were 6150,000 persons released after serving their sentences, indicating that the connection rate of persons released after serving their sentences showed a slight downward trend. The author also combed and analyzed the overall connection rate of persons released after serving their sentences in recent years, and the results were shown in Figure 3.

As can be seen from Figure 3, the overall connection rate of those released from prison in 2011 and 2015 showed a downward trend, indicating that the growth rate of the number of those who have been connected was lower than that of the total number of those released from prison [14]. As the starting point of follow-up resettlement, assistance, and education, the overall connection rate is declining, and the gap between the number of people who have been connected and the total number of released people is widening, which indicates that more released people are not under the control of the public security and judicial organs, which will inevitably affect the follow-up protection work but also bring difficulties to crime governance.

The article "Paradigm and Path of Released Prisoners' Rights of Rehabilitation from the Perspective of Social Governance" was retracted in 2023. Reasons: unreliable results or conclusions; concerns about the data; concerns about the peer review; concerns about the citations.

The policy of “mandatory transfer” should be implemented for key help and education recipients, that is, the key help and education recipients must be transferred out of prison by relevant organizations or units, so as to prevent them from directly entering society and escaping control. However, from the practice in 2013 and 2015, the connection of key help and education objects and the implementation of control measures are shown in Table 1

As can be seen from Table 1, in terms of connection, the connection rate of key help and education objects in China has not reached 100% in recent years, and 10% and 20% of people are still not connected every year. According to the implementation rate of control measures for key objects of help and education, nearly half of them are still outside the control of public security and judicial organs [15]. Moreover, the implementation rate calculated by the author is based on the actual number of connections. If calculated according to the number of connections, the implementation rate may be lower.

In order to ensure that the released prisoners do not go out of control when they transition from prison to society, the social protection work for them needs to follow certain procedures and the active cooperation of relevant departments [16]. This article learned from the investigation of a county Justice Bureau that at present, in order to strengthen the information database construction of prisoners and better carry out resettlement, help, and education work, the Ministry of Justice has developed an information management system for released prisoners. The system connects the judicial administration department and the public security department with special client interfaces accordingly to carry out standardized management of the connection placement, help, and education work. The specific protection workflow is illustrated in Figure 4.

As can be seen from Figure 4, the application of an information management system for released prisoners ensures the docking of information about prisoners among various connecting subjects. But, in practice, the application of the information platform is only connected in form, while the implementation of the essence is restricted by a variety of factors in the subject of protection. For example, in the information verification of prisoners and the follow-up of help and education measures, it is difficult for the grassroots judicial administrative organs to share the strength to implement this work.

The article "Paradigm and Path of Released Prisoners' Rights of Rehabilitation from the Perspective of Social Governance" was retracted in 2023. Reasons: unreliable results or conclusions; concerns about the data; concerns about the peer review; concerns about the citations.

#### 3.2.2. Resettlement of Persons Released after Serving Their Sentences

In 2015, a total of 773,000 released persons were resettled, with the resettlement rate accounting for 95.8% of the connected population. The author summarized the overall resettlement situation of released persons in China from 2011 to 2015, as shown in Figure 5.

As can be seen from Figure 5, the settlement rate shows an increasing trend [16]. It can be inferred from the previous article that the total number of people released after serving their sentences is increasing. According to the above connection rate, 697,000 people were relocated in China in 2014, and 544,000 people were relocated in 2013, which means that the total number of resettlement is expanding, indicating that the overall resettlement of people released after serving their sentences is developing toward a better situation [17].

Take the resettlement situation of released prisoners in 2015 as an example for specific analysis (as shown in Figure 6). In 2015, 45,000 people were resettled in enterprise resettlement bases, accounting for 5.8% of the total resettlement; The transitional resettlement bases mainly funded by the government resettled 50,200 people, accounting for 0.7%; 380,400, or 49.2%, were designated as responsible farmland. A total of 2,000, or 0.3%, were assigned to public welfare jobs. A total of 45,100, or 5.8%, started their own businesses; 67,800, or 8.8%, are self-employed. Enterprises and economic entities created 44,400 jobs, accounting for 5.7% of the total, while 183,100, or 23.7%, were employed by other means [18].

#### 3.2.3. Conditions of Help and Education for Those Released after Serving Their Sentences

In order to facilitate the smooth transition of released prisoners to society, the nonmandatory guidance and assistance education and management activities for this group in the process of rehabilitation are not only a guarantee of rights at the institutional level but also a dynamic and all-round protection measure [19]. With the efforts of all sectors of society, China's help and education work has achieved good results. In 2015, there were about 801,800 people helping and teaching, with the help and education rate reaching 99.4%. The author made a summary of the help and education situation of released prisoners from 2011 to 2015, as shown in Figure 7 below, with the help and education rate above 95%.

The article "Paradigm and Path of Released Prisoners' Rights of Rehabilitation from the Perspective of Social Governance" was retracted in 2023. Reasons: unreliable results or conclusions; concerns about the data; concerns about the peer review; concerns about the citations.

While we have made great achievements, we should also note the inadequacies. The number of people without help or education still accounts for a considerable proportion. In 2015, more than 1.362 million people were released after serving their sentences, and more than 5.309 million were in the process of receiving help and education. There is still a big gap between the number of people who received help and education, and the work of helping and education needs to be further strengthened.

Take the implementation of social assistance and preferential policies for those released after serving their sentences in 2015 as an example (see Figure 8); the specific situation of help and education in China is analyzed. In 2015, 94,700 people received social assistance, including 10,200, or 10.8%, who received subsistence allowances. A total of 0.09 million, or 0.9%, were provided for in extreme poverty. Medical assistance was provided to 40,800 people, or 5.1% of the total; housing assistance was provided to 10,000 people, or 1.1% of the total. A total of 14,200, or 15.0%, received temporary assistance; 9,400, or 9.9%, were registered as unemployed; skills training was provided to 28,400, accounting for 30.0%; 24,800, or 26.2%, were recommended for employment [20].

As can be seen from Figure 8, the assistance to released persons is mainly provided in three ways, namely, recommending employment through skill training and implementing temporary assistance, with the three accounting for a large proportion of 71.2%, and the implementation of these relief measures needs the support of social forces, while the current help and education work is basically promoted by government departments, and the lack of participation of social member units restricts the development of help and education work [21]. In 2015, of the more than 800,000 people released after serving their sentences, only 94,700 received social assistance, accounting for only 11.7% of the total, and nearly 90% of those still did not receive social assistance.

### 3.3. The Recidivism Situation of People Released after Serving Their Sentences in China

#### 3.3.1. National Statistics on Recidivism

Searching from the website of the National Bureau of Statistics, the changes in the number of prisoners released in recent years are sorted out in Table 2.

As shown in Table 2, the total number of prisoners in our country is increasing. The proportion of recidivism in prisons nationwide has been on the rise from 6.3% in 1984, 8.6% in 1990, 11.1% in 1996, 12.86% in 2003, and 14.8% in 2006.

The article "Paradigm and Path of Released Prisoners' Rights of Rehabilitation from the Perspective of Social Governance" was retracted in 2023. Reasons: unreliable results or conclusions; concerns about the data; concerns about the peer review; concerns about the citations.

#### 3.3.2. Statistics of Recidivism in Prisons of Some Provinces and Cities

Some scholars conducted a survey on recidivism in Fujian province in 2001 and 2005 and finally calculated the proportion of recidivism in all prisoners in the provincial prison system in each year as shown in Table 3 (proportion of recidivism = number of recidivism and number of prisoners).

The number of prisoners is increasing, but the proportion of reoffenders is also increasing. In terms of proportion, the increase rate of recidivism is obviously higher than that of prisoners, showing that the problem of recidivism of released prisoners is becoming more and more serious. The emergence of this phenomenon is not accidental. In the period of social transition, the old social control mechanism is broken, while the new one is not established, which inevitably leaves room for the crime.

#### 3.3.3. The Specific Conditions of Recidivism

In the first half of 2016, the author investigated a prison and conducted a questionnaire survey on 275 recidivism prisoners in the prison [22]. A total of 180 valid questionnaires were collected and analyzed, and the current situation of recidivism was specifically explained from three aspects (Tables 4–6).

According to the statistics in Table 4, the recidivism of released persons is theft, robbery, fraud, and robbery, which accounts for the highest proportion. According to the statistics in Table 5, recidivism is likely to occur at any time after release, and the proportion of recidivism within 5 years is 73.3%, which indicates that recidivism occurs frequently within 5 years after release. At this time, the management and control of released persons should be strengthened. However, it is worth noting that the proportion of reoffenders who have been released after serving their sentences for more than 5 years still accounts for 26.7%. It can be seen that the 5-year period of placement, help, and education is not enough to control reoffenders, and the placement, help, and education work needs long-term follow-up [23]. According to the statistics in Table 6, there is a large difference in the length of sentence for the first crime and the second crime, and the proportion of the sentence for the first crime is less than 5 years is 86.1%. The proportion of those sentenced to less than 3 years for the second offense was 31.1%, 25.6% lower than 56.7% for the first offense. The proportion of those sentenced to 3 to 5 years increased by 20.7% compared to the first time, and the proportion of those sentenced to 5 to 10 years was almost the same as the first time. However, the proportion of those sentenced to more than 10 years increased to 8.4%, an increase of 6.2% compared to the first time, indicating that the second time is more serious than the first time, and the situation of reoffending is worsening.

The article "Paradigm and Path of Released Prisoners' Rights of Rehabilitation from the Perspective of Social Governance" was retracted in 2023. Reasons: unreliable results or conclusions; concerns about the data; concerns about the peer review; concerns about the citations.

## 4. Personal Factors Affecting the Return of Released Prisoners

### 4.1. Personal Conditions of Persons Released after Serving Their Sentences

The personal conditions of released prisoners include biological conditions such as age, gender, citizenship status, occupation, residence, marriage, social class, education level, and other social conditions. The age statistics of reoffenders released from prison are summarized in Table 7. It can be seen that recidivism released from prison was young when they committed their first crime, accounting for 78.3% of them under the age of 35. This age group is in the golden period of employment and the establishment of marriage and family. After the reform of the prison, the number of offenders under the age of 25 drops significantly, and most of them are over the age of 26, and the number of all ages over the age of 26 has increased compared with the first time they committed a crime. Their age often affects their employment opportunities and thus their return.

It can be seen from Table 8 that the educational level of reoffenders is mostly concentrated in junior high school and below, and the educational level is low. Psychological studies show that educational level affects individual cognitive thinking and self-control ability. A higher educational level means better ability to correctly recognize and control themselves. It can be seen from Table 8 that the educational level of reoffenders is mostly concentrated in junior high school and below, and the educational level is low [24]. Psychological studies show that educational level affects individual cognitive thinking and self-control ability. A higher educational level means better ability to correctly recognize and control themselves. For prisoners, when their education level is higher, they are more able to accept new things and have a deeper understanding of their own criminal behaviors.

It can be seen from Table 9 that most of the released recidivists are unmarried. The author analyzes the reasons for their unmarried status. One is that they were not married before and it is difficult for them to find a partner after their release due to their criminal prison experience; the other is that they were married before, but their wife ran away or divorced because of their imprisonment.

As can be seen from Table 10, the proportion of unemployed and migrant workers is larger both before the first crime and when the crime is committed again, and the proportion of unemployed workers when the crime is committed again is larger than before. Faced with the rapidly changing society, released prisoners lack the survival skills to adapt to society, resulting in a jobless state after release, which is very likely to lead to recidivism.

The article "Paradigm and Path of Released Prisoners' Rights of Rehabilitation from the Perspective of Social Governance" was retracted in 2023. Reasons: unreliable results or conclusions; concerns about the data; concerns about the peer review; concerns about the citations.

### 4.2. Countermeasures and Suggestions on the Return of Released Persons to Society

#### 4.2.1. Giving Full Play to the Government's Leading Role

Policy support includes in-prison policy and post-release social policy. For example, prisoners are supported to obtain remuneration through their own labor and use the remuneration for their own social insurance. The main purpose is to satisfy the basic living needs of prisoners after their release from prison and reduce the possibility of recommitting crimes, so as to demonstrate the strength and image of domestic human rights protection work. The social insurance for prisoners is different from that of local people, and there should be some unique principles in its implementation. In terms of capital input, the investment direction is not only a one-time investment such as issuing temporary relief and renting temporary sites but also the establishment of long-term relief funds related to the government's initiative to purchase the services of social nonprofit organizations. With the support of funds, NGOs can better adapt to their work and achieve the desired results.

### 4.3. Strengthen Cooperation between Government Departments

The work of returning to a society for released persons after serving their sentence is carried out in accordance with the way of education in prison. After being released from prison, it is continued by the Justice Bureau, and the Justice Bureau is responsible for the main work of returning to society. This work also needs the cooperation of other departments. There is a requirement and regulation for this work, but there is no specific implementation method and authority for the cooperation as far as the current development situation is concerned. Under the condition that all government departments fulfill their main responsibilities, the government organizes relevant departments to cooperate in the work of returning released prisoners to society. In the system of politics and law, the Bureau of Justice and the prison are the main starting point of the return to society, but the court and procuratorate of the Public Security Bureau are also an important part of the system of politics and law, which can play a great role in the return to society. In addition, it is necessary to cooperate with the civil affairs department, human resources security department, industrial and commercial tax department, urban administration department, and other departments to seek a variety of ways and means to return to social work as far as possible, to provide employment places for those with technical ability, and to provide necessary entrepreneurial help for those who plan to seek their own careers. The government should clarify the scope and rights and responsibilities of cooperation and governance among various departments and strengthen communication and exchanges between departments so that the work of returning released prisoners to society can be carried out effectively under the requirements of the government and achieve practical results.

The article "Paradigm and Path of Released Prisoners' Rights of Rehabilitation from the Perspective of Social Governance" was retracted in 2023. Reasons: unreliable results or conclusions; concerns about the data; concerns about the peer review; concerns about the citations.

### 4.4. The Government Has Strengthened the Security System and Strengthened the Training of Professional Personnel

The return of released persons to social work needs the cooperation of all departments under the leadership of the government. Strengthening the leadership of the government is the premise of cooperative governance, and strengthening the institutional construction is important support. Especially in terms of strengthening the security system for those released after serving their sentences, they should pay more attention to the social assistance system. For example, prison-released people in extreme poverty have been included in the unified management of subsistence allowance families, so as to avoid the situation of having food in prison and being neglected when they return home. Social assistance has been provided to people released from prison in extreme poverty so that they can safely return to society and avoid committing crimes again. At present, the Justice Bureau of some provinceis short of professionals who are engaged in the work of returning released persons to society after serving their sentences. Colleges and universities should set up relevant majors or cooperate with the government to run schools, set up training modes, and especially transport judicial professionals to carry out this work. The government should provide appropriate post-welfare benefits and management system to ensure that professional talents do not lose and ensure professional personnel for the return of released persons to social work.

### 4.5. Deepen Effective Cooperation between the Government and Nongovernmental Organizations

The cooperation between government and nongovernment is deepened because, in some work, nongovernment acts represent the government and can exert the work effect that government organizations cannot achieve. The government plays a guiding role in the reintegration of released persons into society, and a friendly relationship of equality, mutual benefit, and win-win is maintained between the government and nongovernmental organizations. NGOs have a clear role and positioning. With the participation of NGOs, released prisoners can relax their mental attitude, and they will not always remember their identity as criminals in front of community correction officers and police. In front of community workers, they can integrate themselves into the ranks of normal people as soon as possible. There are two important aspects to deepening cooperation between the government and nongovernmental organizations. One is financial support and the other is talent support. First, nongovernmental organizations are nonprofit organizations, which need a lot of financial support when they are in normal operation. It can be said that the government itself and social donations constitute an important part of such funds. Secondly, the participation of nongovernmental organizations needs the support of talents. More support should be given to the staff of nongovernmental organizations to improve their enthusiasm for work. If NGOs are to achieve the desired results, there should be a certain proportion of professionals in the workforce. The participation of professionals in the development of the work can better implement the policy requirements of the government, and the relevant policies of help, education, and assistance issued by the government can be implemented in place. In the work contact with the released persons, professionals can more accurately grasp the ideological status of the released persons and better help solve the difficulties in returning to society so that they can better adapt to society and further work and life.

The article "Paradigm and Path of Released Prisoners' Rights of Rehabilitation from the Perspective of Social Governance" was retracted in 2023. Reasons: unreliable results or conclusions; concerns about the data; concerns about the peer review; concerns about the citations.

The participation of the whole society is actually the participation of the people. Many government departments have set up public welfare posts, and grid workers are set up in community streets. Most of them are residents who have worked and lived in community streets for a long time so that they can understand the actual situation and carry out their work conveniently. For the work of releasing people back to society, the government involves the public in the work by setting up community correction support officers and grid-like members for public interest work to break the mystery and isolation of released people. Adopting a community street support model will allow the released group to integrate as soon as possible. In addition to public interest jobs, a pool of people returning to society can be created. The construction of a talent pool not only can help those released after serving their sentences in legal employment and other professional knowledge but also provide psychological guidance and guidance in life experience, so as to help those released after serving their sentences to take the right path back to society. The talent pool can help government organizations or nongovernmental organizations in the community when needed so that the whole society can participate in the reintegration of ex-prisoners into society. In order to create a good social environment, it is necessary for the government, civil organizations, and the whole society to participate in the work of returning released persons to society in China. It is conducive to mobilizing their enthusiasm to return to society, increasing social care for them to a reasonable extent, and ensuring that those released from prison feel the society from the bottom of their hearts. They can feel the tolerance and warmth of this big family and ensure that they can truly participate in the governance and operation of the whole society on an equal footing.

The article "Paradigm and Path of Released Prisoners' Rights of Rehabilitation from the Perspective of Social Governance" was retracted in 2023. Reasons: unreliable results or conclusions; concerns about the data; concerns about the peer review; concerns about the citations.

## 5. Conclusion

It is of great significance for the country, the society, the family, and the individual that the released persons return to society. In recent years, the government and society are increasingly concerned about this issue. Through the investigation of the main factors affecting the rehabilitation of the released prisoners and the specific situation of reoffending, it is found that the sentencing period of the first crime and the second crime is quite different. The proportion of those sentenced to less than five years for the first time was 86.1%, and those sentenced to less than 3 years for the second time was 31.1%, which decreased by 56.7% compared to the first time. The proportion of those sentenced to more than 10 years increased by 8.6%, indicating that the second crime is more serious than the first crime. Those released from prison are likely to commit crimes again at any time after rehabilitation, and the proportion of reoffending within 5 years is 73.3%. The proportion of reoffenders who committed crimes for more than 5 years was 26.7%, indicating that the 5-year period after rehabilitation should be taken seriously to reduce the second crime rate.

Therefore, in the long run, the government and nongovernmental organizations, as well as everyone in society, including the released prisoners themselves, play a very important role in the return of released prisoners to social work and are indispensable and important links. It is not appropriate to promote the return of released prisoners to social work in a big way to improve social cognition and acceptance and, to some extent, to improve the social and cultural level of the rehabilitation effect of released prisoners through We-Media publicity. These subtle things really need to be done, and these efforts need an effective and reasonable mechanism to drive long-term development. From the starting point of my research, using the concept of cooperative governance to establish a governance system for the return of released prisoners to society is an effective and sustainable way.

The article "Paradigm and Path of Released Prisoners' Rights of Rehabilitation from the Perspective of Social Governance" was retracted in 2023. Reasons: unreliable results or conclusions; concerns about the data; concerns about the peer review; concerns about the citations.

## Figures and Tables

**Figure 1:** A new system of social governance.

**Figure 2:** Chart of changes in the number of people released after serving their sentences during 2011–2025.

**Figure 3:** Chart of changes in the overall cohesion rate of those released after serving their sentences during 2011–2015.

**Figure 4:** People released after serving their sentences link up the working process.

**Figure 5:** Chart of changes in the overall resettlement rate of those released after serving their sentences during 2011–2015.

**Figure 6:** The specific resettlement type of persons released after serving their sentences in 2015.

**Figure 7:** Chart of changes in the overall help and education rate of those released after serving their sentences during 2011–2015.

**Figure 8:** Social assistance for released prisoners in 2015.

**Table 1:** Key objects of help and education and the implementation of control measures during 2013–2015.

Year	The actual cohesion	Should join	Convergence rate (%)	Implement control measures	Implementation rate (%)
2015	43,500	47,300	88.7	22,400	49.3
2014	34,600	31,000	88.5	20,800	65.6
2013	38,400	30,000	19.1	13,500	52.6

**Table 2:** Changes in the number of prisoners released during 2006–2013.

	2013	2012	2011	2010	2009	2008	2007	2006
Number of people in prison at the beginning of the year/man-time	1,665,963	1,641,931	1,656,773	1,646,653	1,623,394	1,589,212	1,566,839	1,565,621
Number of people in prison at the end of the year/man-time	1,698,541	1,657,863	1,642,931	1,656,459	1,646,593	1,623,394	1,589,210	1,566,839
Rehabilitation personnel	325,479	395,017	403,106	391,270	387,172	378,493	363,765	340,784

**Table 3:** Prisoners in the Fujian prison system during 2001–2005.

Year	Inmates	Repeat the number	Recidivism rate (%)
2001	51,381	5,436	11.8
2002	53,314	6,151	12.4
2003	43,870	6,424	10.4
2004	54,629	8,232	12.9
2005	55,795	7,854	12.1

**Table 4:** The specific types of reoffending of released persons.

Recidivism type	Theft	Robbery	Loot	Fraud	Injure or kill with intent	Rape	Extortion	Provoke troubles
Number	73	32	25	21	15	15	6	5
Percentage (%)	38.4	11.7	7.9	12.7	7.7	5.6	3.7	1.8

**Table 5:** The time between release and reoffending.

Time interval between recidivism	Number of people	Percentage (%)
Less than 1 year (inclusive)	37	20.4
1–3 years (including 3 years)	46	28.7
3–5 years (including 5 years)	39	21.2
Over 5 years	38	25.7

The article "Paradigm and Path of Released Prisoners' Rights of Rehabilitation from the Perspective of Social Governance" was retracted in 2023. Reasons: unreliable results or conclusions; concerns about the data; concerns about the peer review; concerns about the citations.

**Table 6:** Comparison of length of sentence for first and second offenses.

	The period of sentencing for the first offense		Sentence period for a second offense	
	Number	Percentage (%)	Number	Percentage (%)
Less than 3 years	104	55.7	65	32.1
3–5 years (including 5 years)	45	28.4	83	51.1
5–10 years (including 10 years)	19	12.7	16	9.4
More than 10 years (including life suspension)	4	2.2	14	8.4

**Table 7:** Comparison of the age of the released recidivism.

	First offense		Reoffense	
	Number	Percentage (%)	Number	Percentage (%)
Under 18	42	17.9	10	7
18–25 years old	56	35.2	35	15
26–35 years old	41	22.1	76	36.5
36–45 years old	15	13.9	45	19
46–55 years old	10	6	23	6.2
Over 56 years old	7	1.8	8	5

**Table 8:** Cultural conditions of reoffenders released from prison.

Standard of culture	Number of people	Percentage (%)
Primary or below	64	32.1
Junior high school	68	34.3
Senior high school	28	11
Junior college or above	9	6.6

**Table 9:** Marital status of reoffenders released from prison.

Marital status after release from prison	Number of people	Percentage (%)
Married (i.e., in a continuing state of marriage)	68	34.3
Unmarried (including divorced and widowed)	101	65.7

**Table 10:** Occupational status of reoffenders released from prison.

	First offense		Reoffense	
	Number	Percentage (%)	Number	Percentage (%)
Unemployed	62	39	84	45.2
Peasant worker	59	23.3	48	26.2
Individual household/private entrepreneur	16	7.3	20	11.7
A state official such as a civil servant	5	3.2	0	0
Others	28	15.2	24	12.9

## Data Availability

The labeled data set used to support the findings of this study can be obtained from the author upon request.
